# Clinical Acupoint Selection for the Treatment of Functional Constipation by Massage and Acupuncture Based on Smart Medical Big Data Analysis

**DOI:** 10.1155/2021/9930412

**Published:** 2021-07-16

**Authors:** Fengzhi Sun, Zhuolin Liu, Wanli Zhang

**Affiliations:** ^1^Chinese Massage Department, The Affiliated Hospital of Shandong University of TCM, Jinan 250014, Shandong, China; ^2^Medical Department, Jinan Children's Welfare Center, Jinan 250013, Shandong, China

## Abstract

With the development of society and economy, people's lifestyle and eating habits have undergone great changes, such as spending a long time behind desks, sitting for a long time, drinking and staying up late, and emotional depression; functional constipation, a disease of the digestive system, has changed. It is extremely common, and the age of onset is gradually decreasing. The development of the medical and health industry is also accompanied by the rapid development of technologies such as the Internet of Things, big data, and artificial intelligence, which penetrates into all aspects of the medical and health field and has entered the stage of smart medical care. This article proposes a study on the clinical acupoint selection rules of massage and acupuncture treatment of functional constipation based on smart medical big data analysis. This article adopts a variety of methods such as literature data method and experimental research method to carry out related theoretical research and promotion of massage and acupuncture treatment under the background of smart medical big data and design a clinical experiment of massage and acupuncture treatment based on big data analysis for functional constipation. The advantages of big data algorithms, the law of selecting acupoints in massage and acupuncture treatment, and the comparison of CCS symptom score and PAC-QOL score are analyzed. From the frequency of acupuncture treatment of functional constipation, the top 5 acupoints are Tianshu, Shangjuxu, Dachangshu, Zusanli, and Zhigou. In this paper, the total effective rate of treatment in the experimental group reached 96.56%, while the total effective rate of treatment in the control group was only 75.02%. Tuina and acupuncture treatment of functional constipation has a good therapeutic effect and is worthy of extensive clinical application.

## 1. Introduction

The times are advancing, and people's living habits and work styles are also diversified, such as spending a long time behind desks, sedentary activities, alcoholism and staying up late, and emotional depression; functional constipation, a disease of the digestive system, has become extremely common, and the age of onset is decreasing gradually. Functional constipation (FC) is a group of syndromes with main symptoms of significantly reduced bowel frequency, dry and hard stool, difficulty in defecation, and incomplete defecation after defecation, and organic diseases have been excluded through various examinations. According to epidemiological data, the prevalence of functional constipation is higher among the elderly, female, nonwhite, low-income, and low-education people, and the incidence rate is 10%–15% in European and American countries.

The cause of functional constipation is not clear in modern medicine, but it is related to many factors. Through the examination of intestinal dynamics, histopathology, X-ray, electrophysiology, and so forth, we found that there are more than 100 types in the 7 categories of diet changes, poor bowel habits, genetic factors, and mental and psychological factors. In terms of treatment, laxatives are the mainstay. In recent years, there have been biofeedback therapy, colon hydrotherapy, microecological preparations, psychological counseling treatment, and so forth. In severe cases, surgical treatment is required. Functional constipation not only reduces the quality of life but also is often accompanied by other diseases, such as colitis, myocardial infarction, hemorrhoids, hypertension, colonic malformations, cerebral hemorrhage, IBS, and colon cancer. With the rapid development of information technology in the medical industry, smart medical care has become the focus of widespread attention at home and abroad. Smart medical care plays an important role in alleviating doctor-patient conflicts caused by information asymmetry and regional health differences caused by irrational allocation of medical resources, as well as improving the level of medical services.

In the work of Kim B., since the rapid spread of the Internet of Things as a new communication mode, people have conducted a lot of research on various applications of the Internet of Things. In particular, people's interest in smart medical systems is increasing day by day. In an intelligent medical system, a large number of medical devices are distributed in popular areas such as stations and medical centers. This high-density distribution of medical devices will cause serious degradation of communication performance, which is called a coexistence problem. When the intelligent medical system has coexistence problems, it may not be able to guarantee the reliable transmission of the patient's biological information, endangering the patient's life safety. Therefore, the coexistence problem in the intelligent medical system must be solved. He proposed a distributed coexistence mitigation scheme for intelligent medical systems based on the Internet of Things, which can dynamically avoid interference in the case of coexistence and ensure reliable communication. In order to evaluate the performance of the proposed scheme, a lot of simulations were conducted by comparison with IEEE802.15.4. But his experimental data is not complete, and the control variable factors are not standard [1]. Wojtyniak and Szajewska updated the 2010 systematic review on the efficacy of probiotics in the treatment of constipation in children. As of February 2017, randomized controlled trials (RCTs) in children without language restrictions were searched in the MEDLINE, Embase, and Cochrane Library databases, clinical trial registration centers, and reference lists of included studies. According to the researcher's definition, the main outcome indicator is the success rate of treatment. They included 7 randomized controlled trials with a total of 515 participants. The included trials are heterogeneous in terms of study population, probiotic strains, dosage, study duration, and follow-up. The combined results of two randomized controlled trials show that in terms of treatment success rate. Other probiotics are only studied in a single trial. Although some probiotic strains have a certain effect on the frequency of bowel movements, none of the probiotics have a beneficial effect on the frequency of fecal incontinence [2]. Karabudak et al.'s study aims to determine the relationship between functional constipation and lifestyle, eating habits, and nutritional status in young people. Karabudak et al.'s study was conducted among 825 young people between 20 and 24 years of age in Ankara. Constipation was assessed by self-report and Rome III criteria. The frequency of food, beverage consumption, and fluid intake were investigated, and anthropometric measurements (weight and height) were evaluated. Concise physical activity assessment tools were used to assess physical activity. Participants reported that they were constipated, not constipated, and sometimes constipated at 7.8%, 39.6%, and 53.6%, respectively. These ratios are different from those obtained using the Rome III criteria: 51.3% with constipation and 48.7% without constipation. The female constipation rate (54.4%) is higher than that of males (44.8%). Their experimental results do not well show the correlation between the factors, and there is a lack of corresponding data conclusion analysis [3].

The innovations of this article are as follows: (1) It combines theoretical analysis with practical analysis, fully applies theoretical foundations in practice, and applies smart medical big data analysis in the treatment of functional constipation; (2) qualitative research and quantitative research are similar; and, in combination, there are both data analysis and qualitative content analysis.

## 2. The Research Method of Clinical Acupoint Selection Rules for the Treatment of Functional Constipation with Massage and Acupuncture Based on Big Data of Smart Medical Care

### 2.1. Smart Medical Care

#### 2.1.1. Smart Medical Care Provides a New Direction for the Construction of “Healthy China”

With the rapid development of China's economy, people's attention to health has gradually changed from disease treatment and control development to disease prevention and health management [4]. The Chinese government has always attached great importance to people's health and made a series of major decisions and deployments. After many rounds of medical and health system reforms, China's medical and health system is not perfect, and the irrational allocation of resources between regions still exists [5]. The construction of medical informatization is one of the important guarantees of the “Healthy China” strategy [6]. In the process of structural reform of the medical and health supply side, the introduction of technological innovation is the general trend. Under the smart mode, existing resources can be fully utilized to relieve the pressure of population, economy, technology, and so forth, adjust the contradiction between supply and demand, solve the tension between doctors and patients, and alleviate the reality question [7].

#### 2.1.2. Smart Healthcare Has Become an Important Means to Promote the Development of Medical Informatization

As people's demand for basic medical services continues to increase, information technology has gradually received attention in medical institutions. In the late 1970s, the interdisciplinary “medical informatics” was derived, marking the formal integration of information technology into the medical field [8]. The development of medical informatization has gone through four stages: (1) The digital medical stage began in the early 1980s. With the popularization of computer applications, medical institutions have gradually realized the necessity and need to combine computer technology with the medical and health industry. Practicality [9], by replacing part of manual operation with small software to assist daily work, the transition of medical informationization from nothing to something has been realized. (2) In the local area network medical treatment stage, starting from the late 1980s, with the advancement of software and material technology [10], the operators of medical institutions gradually developed the hospital information system, which was used as an important tool for medical information management. The complete set is developed based on this. It manages the various parts of the system [11]. Commonly used working software and database systems such as HIS, PACS, and LIS send medical information to hospitals in the local network [12]. (3) At the stage of Internet medical treatment, the medical and health industry began to explore regional cooperation in medical information, such as telemedicine, online self-health consultation, electronic prescription, and other functions, which realized the information exchange and sharing between medical institutions [13]. (4) The stage of smart medical care began in the early 21st century. Due to the communication and interaction among patients, medical personnel, medical institutions, and medical devices, the use of the most advanced Internet, big data, artificial intelligence, and other technologies was emphasized [14]. The generation of information is inseparable from the rapid development of medical and health departments [15]. Smart medicine has huge application potential in the process of medical management, and it has become an important means to promote the development of medical information.

#### 2.1.3. Smart Healthcare Has Become a Connotative Force That Promotes the Positive Development of the Doctor-Patient Relationship

In recent years, the doctor-patient relationship has become increasingly “freezing,” and the violent environment has caused panic and indignation among medical staff and all walks of life. The core of improving doctor-patient friendliness is to optimize the hospital's medical treatment process and communication channels. With the rapid development of information technology [16, 17], smart medical care provides new perspectives and tools for improving the medical experience, and the online information interaction model provides doctor-patient communication. A new platform effectively solves the problem of information asymmetry between doctors and patients, thereby promoting the positive development of doctor-patient relations [18].

The main research areas of smart medical care are the following: (1) Research on technological innovation. From the medical service application model, the medical management application model, and the medical device management application model, the medical Internet of Things application model is researched, from the big data through the innovative medical technology, to improve the service level, as well as from the big data to innovate the medical service supply chain management [19]. (2) Research on factors affecting smart medical care. At present, there is insufficient empirical research on the impact of smart medical system applications on patient satisfaction [20]. Understanding the habit of using information systems and the complexity of the diagnosis and treatment process, the intention of adopting innovative products will increase doctors' satisfaction with their work. (3) Research on smart medical service model [21]. It introduces the core technology and market development of smart wearable devices from the technical layer, perception layer, and service layer and points out that the future smart wearable devices will use sensors to collect data and upload it to the cloud, so as to customize services for users. (4) Research on the privacy of smart medical users. The discussion of data security and privacy is proposed for medical wearable devices. Through the analysis of the results of the questionnaire, it is found that users lack the awareness of confidentiality and the concept of respecting others' privacy is poor [22, 23], and corresponding protection strategies are proposed.

### 2.2. Big Data

In recent years, the national economy has developed rapidly, and the country's investment in the medical field has gradually increased. With the continuous expansion of the scale of hospitals, how to effectively improve the level of hospital management has become the key point of medical services [24]. The rapid expansion of hospital scale has brought about the generation and accumulation of massive medical data. The existing information management system of hospital institutions relies on traditional data warehousing and only provides storage and query statistics services for these medical data [25]. Not only does the unreasonable data storage of these huge amounts of medical data consume huge resources in the hospital but also the lack of data analysis and prediction services makes it impossible to dig out the data value behind these medical big data [26], which leads to the level of medical services and management to not be effectively promoted. With the increasing maturity of big-data-related technologies and the continuous improvement of hospital construction, the use of big-data-related technologies to process hospital medical data, analyze and predict the data, and provide references for the development of hospitals has received more and more attention.

The application of big data in the domestic medical field is mainly divided into the following aspects:

1. Electronic management of medical treatment data: medical treatment data mainly includes various indicators such as medical test results, patient's medical history, patient's family medical history, and patient's information [27]. The amount of these data is very large, and the operation of data storage and data processing is very difficult. Big data technology can be used to quickly analyze and process medical data.
2. Health prediction: establish a health prediction model based on the statistics of wearable devices such as smart bracelets and smart watches. These wearable statistical devices continuously collect data and store the data in the cloud to monitor the health of patients in real time. These big data are used in the prediction and analysis of various diseases.
3. Clinical diagnosis: through the storage of massive medical images, including nuclear magnetic resonance images, ultrasound images, and X-ray images, data mining and deep learning are carried out. By training the model to diagnose the film, it assists the doctor to complete the clinical diagnosis decision and improves the efficiency of the doctor's work.
4. Drug research and development: use the big data of each drug index to carry out data modeling analysis, predict the clinical trial results of the drug, and reduce the time spent in the clinical trial stage of the drug. Pharmaceutical manufacturers can produce drugs with a higher cure rate through modeling and analysis of drug big data and shorten the time required for the entire process from drug development to market launch.

The application of big data in other fields is mainly divided into the following aspects.

#### 2.2.1. Smart City

Smart cities use advanced information and communication technologies to conduct statistical analysis on various main indicators and use city operation forecasts as indicators of development trends to accurately, intelligently, and quickly respond to various needs for urban services. The essence of a smart city is the smart management and operation of the city. The core of the smart city lies in the prediction of the trend, and the prediction of the trend needs to be based on the forecast analysis of massive data. The data sample size must be sufficient to ensure the accuracy of trend prediction, that is, the degree of intelligence of smart cities. Therefore, the development of smart cities is inseparable from big data technology.

#### 2.2.2. Virtual Reality

Virtual reality constructs a simulation system that can use a computer to combine multiple information sources to experience the virtual world of dynamic scenes interacting with users. The user can create a virtual world to simulate the physical actions of the system, and the user can be immersed in the virtual environment. The combination of big data and virtual reality is bound to promote the development and application of virtual reality.

#### 2.2.3. Artificial Intelligence

Artificial intelligence is often referred to as AI, which studies theoretical methods and technical systems applied to anthropology and expands anthropology and technical sciences. Artificial intelligence is mainly about simulation training models, which need to be imported into massive amounts of data to achieve the effect of high-end simulation. The development of AI is closely integrated with big data.

### 2.3. Functional Constipation

Constipation will be on its own and will also appear in the course of various acute and chronic diseases. Functional constipation is caused by changes in lifestyle, bad bowel habits, emotional problems, or disorderly taking drugs, and organic diseases such as irritable bowel syndrome are excluded. Many classic literatures in the past had rich records on the etiology and pathogenesis of constipation, and the main reasons are that the stomach and fu organs are unbalanced, the heat in the stomach is flaming, and the spleen meridian dampness internal resistance interferes with the normal operation of the air machine, resulting in difficulty in excretion of stool; the lung qi is stagnant. Failure to obstruct, together with the up-and-down imbalance of the stomach and qi, will cause difficulty in the stool; if the heart is blazing, it will cause the heat and evil to torture the yin fluid, so the intestines are insufficiently moisturized, and eventually the stool will be blocked.

#### 2.3.1. Classification of Functional Constipation

Contemporary physicians are based on the classification of ancient physicians, combined with their own clinical experience, and take the etiology and viscera differentiation as the main guidance for classification. In both, constipation is divided into two categories, Exact Secretion and Deficiency Secretion, as follows: Exact Secretion contains cold secretion, heat secretion, and Qi secretion, and Deficiency Secretion contains yin deficiency secretion, yang deficiency secretion, qi deficiency secretion, and blood deficiency secretion.

#### 2.3.2. Treatment Methods

Traditional Chinese medicine treats functional constipation according to the etiology and pathogenesis of patients with constipation and then treats them accordingly. Although the general principle requires dredging and diarrhea, the amount of laxatives used must vary from person to person and must not be used in large quantities.” In the books on constipation in the past dynasties, it is widely involved in the treatment of the disease, the prescriptions, and the treatment, and the prevention and contraindications are recorded. The treatment methods are mainly external treatment and internal treatment.

#### 2.3.3. Mechanism of Functional Constipation

Defecation is one of human physiological activities; it is a very complex physiological process in the digestive tract. It is a complex reflex activity coordinated by a variety of factors. It is controlled and innervated by the brain and involves the use of nerves and muscles. If there is an abnormality in a certain link of this physiological reflex, which leads to difficulty in defecation, reduced defecation frequency, dry stool, and/or incomplete defecation, it is constipation, and constipation is a clinically very common digestive tract disease, and it is also the most common. It is also one of the symptoms that greatly affect the quality of life. The causes of constipation are extremely complex and can be divided into two types: organic and functional. The causes of organic constipation are colorectal space-occupying lesions, stenosis, obstruction or inflammation, and so forth, which require surgical treatment. Organic constipation also includes secondary constipation, such as diseases of the digestive system (anal fissure, embolic internal hemorrhoids, intestinal tumors, etc.), neurological diseases (stroke, spinal injury, etc.), endocrine system diseases (obesity), and diabetes. Except for constipation caused by organic diseases, metabolic disorders, structural abnormalities, and irritable bowel syndrome, the stool is functional constipation. According to colon dynamics, functional constipation can be divided into three types: slow transit constipation (STC), outlet obstructive constipation (OOC), and mixed constipation (MIX).

The specific mechanism of functional constipation is currently unclear, but it is related to many factors. In recent years, many methods have been used to study the mechanism of functional constipation, such as bowel dynamics, histopathology, radiography, and electrophysiology, and it was found that there are 7 categories and more than 100 kinds, clarifying some of the pathophysiological basis of functional constipation from the aspects of morphology and function.

#### 2.3.4. Influence of Diet Structure

With the progress of modern life, people's requirements for food continue to increase, and there are more and more refined and protein foods. At the same time, the plant fiber contained in the food has been significantly reduced, the amount of feces is insufficient, and the result has been weakened. The normal physiological stimulation of the digestive tract and the regulatory functions of the cerebral cortex and the nerve center are not stimulated, the stomach-colon reflex is also weakened, the peristalsis slows down, and the normal flora in the intestine is also affected, and its fermentation effect is greatly reduced, causing constipation.

### 2.4. Support Vector Machine Algorithm

SVM algorithm models such as linear regression, stepwise regression, and hierarchical regression cannot fully reflect the relationship between the feature vector and the dependent variable. But the optimal hyperplane mapping relationship constructed by SVM can get better results than traditional measurement methods to a certain extent. Under the analysis of smart medical big data, the optimal hyperplane mapping can be used to divide the data space very well, which greatly simplifies the classification and regression of medical data.

Set the separation hyperplane *σ*^*P*^*x*+*b*=0 to correctly separate the sample set {(*u*_*i*_, *t*_*i*_), *i*=1, *K*, *N*}; namely,

(1) $$\begin{array}{c} \left\{\begin{array}{c} \sigma^{P}x+b\geq 1,\text{when}t_{i}=+1,\\ \sigma^{P}x+b\leq -1,\text{when}t_{i}=-1. \end{array}\right. \end{array}$$

Then, the “margin” of the separating hyperplane is defined as

(2) $$\begin{array}{c} \text{margin}=u_{+}+u_{-}, \end{array}$$

where

(3) $$\begin{array}{c} \left\{\begin{array}{c} u_{+}=\underset{i,j=1}{\min}\left\{\frac{\left(\sigma^{P}x_{i}+b\right)}{\left\|\sigma \right\|}\right\},\\ u_{-}=\underset{i,j=1}{\min}\left\{\frac{\left(\sigma^{P}x_{i}+b\right)}{\left\|\sigma \right\|}\right\}. \end{array}\right. \end{array}$$

The “margin” of the separating hyperplane defined in this paper is the sum of the shortest distances from the two types of sample points of different categories to the hyperplane. The larger the “margin” of the obtained separation hyperplane, the stronger the ability to classify samples. Linear SVM is to require the optimal classification hyperplane, that is, the requirement *σ*^*P*^*x*+*b*=0, where *σ* is the solution of the following convex quadratic programming (Q1):

(4) $$\begin{array}{c} \left(\text{Q}1\right)=\left\{\begin{array}{c} \min\frac{1}{2}\sigma^{P}\sigma ,\\ s.u:t_{i}\left(\sigma^{P}x_{i}+b\right)\geq 1,\;i=1,K,N. \end{array}\right. \end{array}$$

Lagrangian function is

(5) $$\begin{array}{c} R\left(\sigma ,b,a\right)=\frac{1}{2}\;\sigma^{P}\sigma -\sum_{i=1}^{N}a_{i}\left[t_{i}\left(\sigma^{P}x_{i}+b\right)-1\right], \end{array}$$

making

(6) $$\begin{array}{c} \frac{\partial R}{\partial \sigma }=0\Rightarrow \sigma =\sum_{i=1}^{N}a_{i}t_{i}x_{i},\\ \frac{\partial R}{\partial b}=0\Rightarrow \sum_{i=1}^{N}a_{i}y_{i}=0,\\ \frac{\partial R}{\partial \alpha_{i}}=0\Rightarrow a_{i}\left[t_{i}\left(\sigma^{P}x_{i}+b\right)-1\right]=0,i=1,K,N. \end{array}$$

Therefore, the KKT condition of (Q1) is composed of the above three equations and the original constraints. Since (Q1) is a convex quadratic programming, the KKT condition is a sufficient and necessary condition for the solution set of (Q1). Then bring it into the dual program (Q2) obtained in (Q1):

(7) $$\begin{array}{c} \left(\text{Q}2\right)=\left\{\begin{array}{c} \underset{\text{s.t.}}{\max}\sum_{i=1}^{N}\alpha_{i}-\frac{1}{2}\sum_{i=1}^{N}\sum_{j=1}^{N}a_{i}a_{j}y_{i}y_{j}x_{i}^{T}x_{j},\\ a_{i}\geq 0,\;i=1,K,N*\sum_{i=1}^{N}a_{i}y_{i}=0. \end{array}\right. \end{array}$$

Suppose that *a*^*∗*^ is the solution of (Q2); then the optimal separation hyperplane obtained by SVM is

(8) $$\begin{array}{c} {\left(\sigma^{*}\right)}^{P}x+b^{*}=0, \end{array}$$

where

(9) $$\begin{array}{c} \sigma^{*}=\sum_{i=1}^{N}a_{i}^{*}y_{i}x_{i}. \end{array}$$

Constraints *b*^*∗*^ must meet the following conditions:

(10) $$\begin{array}{c} \alpha_{i}\left[y_{i}\left(\sigma^{P}x_{i}+b\right)-1\right]=0,i=1,K,N. \end{array}$$

If *α*_*k*_^*∗*^ ≠ 0, then

(11) $$\begin{array}{c} t_{k}\left(\sigma^{P}x_{k}+b\right)-1=0. \end{array}$$

Get

(12) $$\begin{array}{c} b^{*}=t_{k}-{\left(\sigma^{*}\right)}^{P}x_{k}. \end{array}$$

In order to comprehensively evaluate the performance of the proposed model, this article uses accuracy, recall, and *F*1 to evaluate the methods involved. The calculation method of each indicator is as follows:

(13) $$\begin{array}{c} \text{accuracy}=\frac{\left(\text{TF}+\text{TN}\right)}{\left(\text{TP}+\text{FP}+\text{TN}+\text{FN}\right)},\\ R=\frac{\text{TP}}{\left(\text{TP}+\text{FN}\right)},\\ F1=\frac{\left(2\times P\times R\right)}{\left(P+R\right)}, \end{array}$$

where *P* is the precision rate, *R* is the recall rate, FP is a false positive case, FN is a false negative case, TP is a true positive case, and TN is a true negative case.

## 3. Research Experiment on Clinical Acupoint Selection Rules of Massage and Acupuncture for Functional Constipation Based on Big Data Analysis of Smart Medical Treatment

### 3.1. Research Objects of Functional Constipation Treatment

The cases in this study are from April 2018 to March 2019. A total of 60 patients in the Tuina Department/Rehabilitation Medicine Department/Pain Department of the Provincial Hospital of Traditional Chinese Medicine met the diagnostic criteria and inclusion criteria of this study. According to the order of selection and the random number table, 60 patients with functional constipation are divided into experimental group (A) and control group (B), and treatment is implemented according to the corresponding number and group. The treatment group (A) had 1 female patient who failed to persist and took laxatives by herself, so it was an excluded case, and the treatment was finally completed in 29 cases; in the control group (B), there was 1 male patient who gave up automatically, and 1 male patient was only treated for 4 weeks; all cases were shedding. In the end, 28 cases met the standard. The focus was on the observation of the clinical efficacy of massage combined with acupuncture in the treatment of functional constipation (spleen and kidney yang deficiency syndrome) and comparing it with the control group of traditional treatment methods. The two groups used the clinical score scale (CCS) for patients with constipation and the quality of life of constipation patients before and after treatment. PAC-QOL scores were used for comparison, focusing on the uniqueness, practicability, and research significance shown in the process of clinical acupuncture and massage treatment of functional constipation (spleen and kidney yang deficiency syndrome). Ideas were chosen and the foundation was laid for their further promotion.

In the experimental group (group A), there were 11 males and 18 females. The youngest was 21 years old, the oldest was 69 years old, and the average age was 42.76 ± 13.86 years. The shortest course of disease was 20 days, and the longest course was 15 years, with average of 2.96 ± 2.13 years; in the control group (group B), there were 12 males and 16 females, age ranged from 22 to 69 years, average age was 43.83 ± 14.09 years, and course of disease was from 22 days to 18 years, with average of 3.04 ± 2.57 years.

### 3.2. Diagnostic Criteria of TCM Syndromes

The main symptom is when feces are stored in the intestines, and then it is difficult to defecate. Secondary symptoms are (1) pale complexion, (2) abdominal distension and pressing, (3) poor appetite, (4) cold limbs, and (5) long and clear urine, in addition to tongue coating and pulse condition: pale and fat tongue, white and greasy coating, and heavy and late pulse. For those with the main symptoms of the above syndromes and any two of the secondary syndromes, the diagnosis can be confirmed by adding tongue coating and pulse condition.

### 3.3. Inclusion Criteria

1. Meet the diagnostic criteria of Rome III functional constipation
2. Those who meet the criteria for yang deficiency of the spleen and kidney in the diagnosis of TCM symptoms
3. Male and female patients between 21 and 69 years of age
4. Before treatment (>2 weeks), except for emergency situations, did not use any drugs to treat constipation, did not receive massage for constipation (>12 weeks), and did not participate in other ongoing clinical researches
5. No obvious abnormality in blood, urine, and stool routine and biochemical examinations, and constipation caused by organic intestinal diseases is excluded through electronic colonoscopy
6. Excluding digestive system (liver, gallbladder, and pancreas) diseases through ultrasound examination
7. Those who have not undergone any anorectal surgery
8. The patient knows and agrees to sign the “Informed Consent,” voluntarily cooperates with treatment research, and returns for consultation

### 3.4. Exclusion Criteria

1. Those who do not meet the above diagnosis or inclusion criteria
2. Patients below the age of 20 and above the age of 70
3. Patients with severe heart, brain, lung, liver, and kidney diseases at the same time, gastrointestinal diseases (Hirschsprung's disease, enteric nerve or muscle disease, inflammatory bowel disease, tumors, etc.), and other diseases that may be involved; patients with systemic disorders of the gastrointestinal tract (spinal cord injury, hypothyroidism, diabetes, connective tissue disease, Parkinson's disease, amyloidosis, etc.)
4. People with infectious diseases, serious skin diseases, skin ulcers/suppurations, and blood diseases
5. Women during pregnancy and lactation
6. Those who have a bad addiction to alcoholism or who are not suitable for drug trial observation
7. Those who have a history of drug or food allergies
8. Constipation caused by taking drugs (calcium channel blockers, psychotropic drugs, opioids, anticholinergic drugs, anticonvulsants, etc.) for the treatment of other diseases
9. People with coagulation dysfunction
10. Fasting and constipation within one month after surgery
11. Those who have a pacemaker
12. Disabled patients prescribed by law (intellectual, psychological, and mental disorders and blindness, deafness, dumbness, physical disability, etc.)
13. Those who have incomplete medical records and have an impact on the efficacy and statistical results

### 3.5. Rejection and Shedding Standards

Those who meet any of the following items will be excluded: (1) choosing other treatment methods during the treatment; (2) adverse events or adverse reactions that occur during the treatment, or the condition continuing to worsen; (3) asked to withdraw from treatment by the attending physician (the effect is not significant, the completion of the questionnaire without cooperation, the withdrawal of the “Informed Consent,” etc.); (4) those whose disease diagnosis is not clear; and (5) those who fail to complete the follow-up consultation in time.

### 3.6. Treatment Methods

The experimental group was treated with massage combined with acupuncture and moxibustion.

Massage techniques included the following: (1) Abdominal manipulation: the patient empties the bladder, takes a supine position, relaxes the entire abdomen, and intends to guard the acupoints being rubbed; and the surgeon stands on the side of the patient and applies the method of rubbing to the center of the abdomen Shu and Guanyuan; the amount of stimulation should be light, 0.5 min per point; the abdomen is rubbed clockwise with palm massage, and the strength in the left lower abdomen is increased appropriately, for about 5 minutes; the surgeon uses the Laogong point to aim at the patient's Shenque point and applies vibration method to make heat penetrate the abdominal cavity. (2) Back operation: the patient takes the prone position, relaxes the lower back, and intends to guard the operated part. The surgeon stands on one side and uses the kneading method or the spine method along both sides of the spine from Ganshu, Pishu to Baliao for round-trip operation, the technique should be light, and the time should be about 5 min; Shenshu, Dachangshu, Ciliao, and Changqiang are pressed and rubbed, and the amount of stimulation should be light, 0.5 min per point. (3) The surgeon stands on the side of the patient, rubbing the shoulders and back, Shenshu, Mingmen, and Baliao, all with the degree of diathermy; rubbing is directly on the back of the Governor Vessel, with the degree of diathermy. (4) The surgeon uses the thumbs of both hands to rub the bilateral branches, Hegu, Zusanli, Shangjuxu, and Taixi for 0.5 min. The above operations were performed once a day, 6 times a week, for a total of 6 weeks of treatment. Key points of operation are as follows: The above treatment techniques require uniformity, softness, longevity, and strong and deep penetration. During treatment, both the surgeon and the patient must be mindful, so as to achieve the best spiritual communication.

For acupuncture therapy, acupunctures Tianshu, Dachangshu, Shangjuxu, Zhigou, and other points for patients with functional constipation, twisting, and purging method for real secrets plus Hegu and Taichong, and Qihai for deficiency of secrets, Zusanli and Guanyuan use the twisting method, 1 time/d, 10 times as 1 course of treatment, and 2 courses of treatment.

The control group was treated with traditional methods only.

### 3.7. Observation Indicators

#### 3.7.1. Symptom Evaluation Index

The Clinical Scoring Scale for Patients with Constipation (CCS) is one of the evaluation indicators of constipation symptoms which has been used by many scholars in recent years. CCS evaluates from eight different aspects, such as the frequency of bowel movements, the degree of effort, the feeling of not being exhausted, abdominal pain, and the type of help needed during defecation. Only the types that need help during defecation are scored by a 3-point method of 0 to 2 points, and other aspects are scored by a 5-point method of 0 to 4 points, and then the items are accumulated in sequence, up to 30 points, and the score is proportional to the severity of the disease.

#### 3.7.2. Main Curative Effect Evaluation Index

In this study, the difference between the scores of CCS and BSFS before and after treatment was compared between groups, and the nimodipine method was used to quantify the efficacy evaluation criteria: (1) Cure: normal bowel movements or recovery to the standard before constipation, with normal symptoms, where the symptom improvement rate is ≥90%; (2) significant effect: significantly improved and close to normal defecation, with most of the other accompanying symptoms absent, with 70% ≤symptom improvement rate <90%; (3) effective: improved bowel movements, with other accompanying symptoms being improved, with 30% ≤symptom improvement rate <70%; (4) ineffective: unimproved or even worsened defecation and other accompanying symptoms, with the symptom improvement rate less than 30%.

After 6 weeks of treatment, the PAC-QOL scores before and after treatment were compared with the total scores according to the four dimensions of PAC-QOL in the treatment group and the control group. The lower the score, the better the effect.

### 3.8. Statistical Methods

SPSS 20.0 statistical software is used for analysis. Measurement data are expressed as mean ± variance (*x* ± *s*), and the data before and after treatment and between groups are compared by paired *t*-test and independent-sample *t*-test; when *P* < 0.05, the difference is statistically significant.

## 4. Analyzing the Clinical Acupoint Selection Rules of Massage and Acupuncture for Functional Constipation Based on Smart Medical Big Data

### 4.1. Comparative Analysis of Big Data Analysis Algorithms

It can be seen from Table 1 and Figure 1 that the improved algorithm performs better than the existing CBA algorithm, CMAR algorithm, and ACSER algorithm in multiple data sets. Through the test on the standard data set, it can be seen that the improved associative classification algorithm has higher classification accuracy and stronger flexibility. Compared with the existing association classification algorithm, the number of rules generated by this algorithm is greatly reduced and the overall efficiency is higher. As a classification algorithm, the prediction accuracy of this algorithm is also very high. Applying the algorithm to the analysis process of the treatment of functional constipation can effectively verify the performance of the algorithm.

### 4.2. The Law of Clinical Acupoint Selection for the Treatment of Functional Constipation by Massage and Acupuncture

Constipation is a common medical disease in traditional Chinese medicine. Traditional Chinese medicine believes that constipation is mostly caused by improper diet, emotional disorders, old age and physical weakness, and feelings of external evil; the disease is mainly in the intestine and is related to the spleen, stomach, lung, liver, kidney, and other visceral dysfunctions; the basic pathogenesis is the conduction dysfunction of the large intestine. Acupuncture and moxibustion treatment of constipation should start from the diseased part and the associated viscera, and the treatment principle is to clear the organs and lead the stagnation.

It can be seen from Table 2 and Figure 2 that the most used acupuncture points for the treatment of constipation in modern acupuncture are Tianshu (526 times), followed by Shangjuxu (366 times), Dachangshu (334 times), Zusanli (328 times), and Zhigou (306 times). Among them, Tianshu acupoint is the most used acupoint and it has a large gap with the value of Shangjuxu in the second place. The values of the acupoints in the 2nd to the 5th place are more balanced, and the value of Qihai in the sixth place is different from Zhigou in the fifth place. Also, the difference between the 6th and 15th positions is more balanced. From the frequency of acupuncture treatment of constipation, the top 5 acupoints are Tianshu, Shangjuxu, Dachangshu, Zusanli, and Zhigou.

According to the “Acupoints Indications,” the acupoints that contain constipation in their main therapeutic effects are Tianshu, Zusanli, Shangjuxu, Xiexi, Dadu, Taibai, Shangqiu, Daheng, Abdomen, Dachangshu, Bladder Shu, Zhongliao, Chengfu, Fuqi, Chuan, Zhibian, Chengshan, Jiaoxin, Zhongzhu, Nanyu, Shangqu, Shiguan, Zhigou, Changqiang, and Zhongwan. Yongquan acupoint mainly treats difficult bowel movement, and Huiyin acupoint mainly treats poor urination and defecation. They are all related to constipation, so they can also be attributed to this type of acupoints that treat constipation. Therefore, there are 27 acupoints that can treat constipation: 8 bladder meridians, 6 kidney meridians, 5 spleen meridians, 4 stomach meridians, 2 Ren channels, 1 Sanjiao meridian, and 1 Du channel.

There are many ways of compatibility of acupoints. The more commonly used methods of compatibility in clinic can be roughly divided into four categories: compatibility by part, compatibility by meridian, compatibility by specific acupoints, and other compatibilities. There is no absolute limit between the various compatibility methods. For example, the original collateral compatibility method belongs to the specific acupoint compatibility, but at the same time it also belongs to the external and internal meridian compatibility method in the meridian compatibility. The calculation method of the association rule is through the adjustment of support and confidence achieved. The support degree represents the probability of two phase sets (phase set X and phase set Y) to appear at the same time, and the confidence degree represents the probability of phase set Y to appear when phase set X appears. Support is used to measure the statistical importance of association rules in the entire data set; confidence is used to measure the credibility of association rules. In the case of constant confidence, the higher the support, the fewer acupoint combinations; in the case of constant support, the higher the confidence, the greater the probability that the two will appear at the same time and the more significant the meaning of compatibility.

The compatibility characteristics of acupuncture prescriptions can be analyzed through the compatibility of acupoints. It can be seen from Table 3 and Figure 3 that the top acupuncture point pattern is Shangjuxu-Tianshu, and its support indicates that the probability that Tianshu and Shangjuxu appear in 619 acupuncture prescriptions at the same time is 56.88%. Degree means that when Shangjuxu appears in the prescription, the probability of Tianshu appearing is 95.92%. From the results of the correlation analysis of acupoint compatibility, it can be seen that the compatibility of acupuncture and moxibustion treatment of constipation with a point compatibility of more than 35% is Shangjuxu and Tianshu, Dachangshu and Tianshu, Zusanli and Tianshu, Zhigou and Tianshu, Shu, Dachangshu, and Shangjuxu, and Dachangshu, Shangjuxu, and Tianshu.

### 4.3. Comparison of the Treatment Score Table between the Experimental Group and the Control Group

It can be seen from Table 4 and Figure 4 that the paired *t*-test was used before and after treatment; when *P* < 0.05, the difference was statistically significant. After treatment, all symptoms in the experimental group (A) except for abdominal pain were higher than those before treatment. *P* < 0.05 indicates significant difference; in the control group (B), all symptoms except for incomplete defecation and abdominal pain were significantly different from those before treatment (*P* < 0.05).

It can be seen from Table 5 and Figure 5 that, after treatment, an independent-sample *t*-test was used within the group; when *P* < 0.05, the difference was statistically significant, indicating that massage and acupuncture treatment of functional constipation accounted for more of the main symptoms of constipation than traditional treatment methods.

It can be seen from Figure 6 and Table 6 that the therapeutic effect of the experimental group is better than that of the control group. The total effective rate of treatment in the experimental group reached 96.56%, while the total effective rate of treatment in the control group was only 75.02%. The difference between the two groups was about 21% improvement rate. In addition, in the control group, there were 7 cases of ineffective treatment, accounting for 25.02%. This shows that traditional treatment methods cannot solve the problems of constipation people well, and the use of massage and acupuncture to treat functional constipation has a good treatment effect.

Figure 7 and Table 7 show the results of the PAC-QOL test. The intragroup comparisons of the two groups before and after acupuncture and massage treatments were performed by paired *t*-test, with *P* < 0.05, indicating that these two treatment options improved the patient's quality of life. The lower the score on the PAC-QOL Quality of Life Scale, the better the quality of the patient. From the point of view of the total score, the experimental group dropped from 84.09 points before treatment to 53.61 points after treatment; the control group dropped from 80.34 points before treatment to 59.61 points, which indicates that the quality of life of the two groups of patients after treatment has been significantly improved.

It can be seen from Figure 8 and Table 8 that the independent-sample *t*-test was used between groups after treatment, with *P* < 0.05, indicating that massage and acupuncture treatment can improve the quality of life of patients more than traditional treatment does. After treatment in the experimental group and the control group, in the comparison of the clinical symptoms of functional constipation (spleen and kidney yang deficiency), the experimental group and the control group both improved to a certain extent. After the comparison of the PAC-QOL rating scale, the patients in the experimental group had better scores than those in the control group in terms of physical condition, mental state, worry, and satisfaction, and all items had *P* < 0.05, indicating that there are statistical differences. Therefore, massage and acupuncture have obvious curative effect in the treatment of functional constipation, and they are worthy of clinical promotion.

## 5. Conclusion

This article mainly studies the clinical acupoint selection rules of massage and acupuncture treatment of functional constipation based on the big data of smart medical treatment. This study mainly chooses the literature method and the experimental research analysis method, and the patients with functional constipation are randomly divided into an experimental group and a control group, under the same treatment cycle, and adopted different treatment methods, evaluated by CCS and PAC-QOL indicators, which were compared and analyzed. To treat functional constipation, this study mainly selected five acupoints, Tianshu, Shangjuxu, Dachangshu, Zusanli, and Zhigou, and used acupuncture and moxibustion in combination with acupoints. The two groups of patients had some improvement after treatment, but the treatment effect of the experimental group is better than that of the control group, and the defecation efficiency and defecation time have been improved. The research method in this paper is worthy of clinical promotion. The main problems in this article are that the number of sample cases selected is too small, and the follow-up investigation of the cases is not carried out. The research on acupuncture points in China is in its infancy, and its development is slower than other aspects of acupuncture and moxibustion. It is hoped that sufficient attention should be given to that in the future research.

## Figures and Tables

**Figure 1:** Algorithm prediction accuracy test results.

**Figure 2:** Frequency of acupuncture and moxibustion treatment of constipation.

**Figure 3:** Correlation analysis of acupoint compatibility.

**Figure 4:** Comparison of the main symptom scores of CCS between the experimental group and the control group before and after treatment.

**Figure 5:** Comparison of the difference scores of the main symptoms of CCS between the experimental group and the control group after treatment.

**Figure 6:** Comparison of efficacy between the two groups after treatment.

**Figure 7:** Comparison of PAC-QOL scores in the two groups before and after treatment.

**Figure 8:** Comparison of PAC-QOL score difference between the two groups after treatment.

**Table 1:** Algorithm prediction accuracy test results.

Data set	Data size	Number of attributes	Number of categories	Forecast accuracy (%)			
				CBA	CMAR	ACSER	Improved algorithm
Breast	698	10	2	96.25	96.43	93.72	96.58
Cleve	313	12	2	82.83	82.28	84.49	83.56
Diabetes	769	9	2	74.45	75.76	77.18	77.23
German	1000	21	2	73.41	74.91	75.01	75.56
Heart	280	14	2	81.86	82.23	82.23	82.91
Horse	359	23	2	82.17	82.62	81.89	82.89
Iris	155	5	4	94.66	94.01	93.34	95.34

**Table 2:** Frequency of acupuncture and moxibustion treatment of constipation.

Serial number	Acupoints	Frequency (times)	Frequency of occurrence (%)
1	Tianshu	526	13.41
2	Shangjuxu	366	9.35
3	Dachangshu	334	8.46
4	Zusanli	328	8.29
5	Branch groove	306	7.78
6	Qihai	143	3.64
7	Guanyuan	138	3.51
8	Zhongwan	134	3.38
9	Pishu	122	3.09
10	Hegu	106	2.68
11	Sanyinjiao	95	2.34
12	Zhaohai	84	2.23
13	Quchi	83	2.11
14	Oyoko	82	2.08
15	Taichong Shenshu	63	1.58

**Table 3:** Correlation analysis of acupoint compatibility.

Serial number	Acupoint mode	Frequency (times)	Support (%)	Confidence (%)
1	Shangjuxu-Tianshu	353	56.88	95.92
2	Dachangshu-Tianshu	312	48.79	90.68
3	Zusanli-Tianshu	310	48.45	91.75
4	Zhigou-Tianshu	286	46.23	93.45
5	Dachangshu-Shangjuxu	223	35.85	66.67
6	Dachangshu, Shangjuxu-Tianshu	218	35.23	98.21
7	Zusanli-Dachangshu	212	34.26	64.82
8	Zhigou-Shangjuxu	211	34.09	69.27
9	Zhigou, Zusanli-Tianshu	166	26.67	95.37
10	Zusanli, Shangjuxu-Dachangshu	145	23.43	68.73
11	Dachangshu, Zusanli, Shangjuxu-Tianshu	143	23.22	99.32
12	Guanyuan-Tianshu	133	21.45	96.37
13	Qihai-Tianshu	131	21.33	92.95
14	Zhongwan-Tianshu	125	20.35	94.85

**Table 4:** Comparison of the main symptom scores of CCS between the experimental group and the control group before and after treatment.

Symptom		Bowel frequency	Struggling to defecate	Feeling of incomplete bowel movements	Stomach ache	Defecation time
Test group (A)	Before therapy	1.42	2.91	2.56	0.94	2.33
	After treatment	0.31	1.19	1.14	0.32	1.15
	Intragroup comparison	*P* < 0.05	*P* < 0.05	*P* < 0.05	*P* > 0.05	*P* < 0.05

Control group (B)	Before therapy	1.38	2.97	2.65	0.91	2.51
	After treatment	0.48	1.88	2.24	0.56	1.38
	Intragroup comparison	*P* < 0.05	*P* < 0.05	*P* > 0.05	*P* > 0.05	*P* < 0.05

**Table 5:** Comparison of the difference scores of the main symptoms of CCS between the experimental group and the control group after treatment.

Symptom	Bowel frequency	Struggling to defecate	Feeling of incomplete bowel movements	Stomach ache	Defecation time
Test group	1.12 ± 0.03	1.82 ± 0.65	1.41 ± 0.67	0.66 ± 0.51	1.16 ± 0.49
Control group	0.91 ± 0.38	1.12 ± 0.52	0.51 ± 0.52	0.33 ± 0.55	0.91 ± 0.62
*T* value	2.126	3.971	5.742	2.425	2.021
*P* value	*P* < 0.05	*P* < 0.05	*P* < 0.05	*P* < 0.05	*P* < 0.05

**Table 6:** Comparison of efficacy between the two groups after treatment.

Group	*N*	Cure	Significantly effective	Effective	Invalid	Total effective rate
Number in the experimental group	29	2	9	17	1	—
Proportion of the experimental group	—	6.71	31.04	58.63	3.45	96.56
Number in the control group	28	1	5	15	7	—
Control ratio	—	3.58	17.86	53.58	25.01	75.02

**Table 7:** Comparison of PAC-QOL scores in the two groups before and after treatment.

Group	Dimension	Before therapy	After treatment	*T* value	*P* value
Test group (A)	Physical	12.63 ± 5.56	8.36 ± 3.36	2.889	*P* < 0.05
	Mental state	21.85 ± 3.64	13.94 ± 4.58	2.812	*P* < 0.05
	Anxiety	32.23 ± 8.71	20.15 ± 4.97	2.843	*P* < 0.05
	Satisfaction	17.68 ± 3.85	11.26 ± 15.56	2.134	*P* < 0.05
	Total score	84.09 ± 22.56	53.63 ± 3.16	3.951	*P* < 0.05

Control group (B)	Physical	13.18 ± 6.14	10.31 ± 3.78	2.311	*P* < 0.05
	Mental state	20.19 ± 6.52	14.42 ± 4.79	2.615	*P* < 0.05
	Anxiety	29.95 ± 4.32	23.85 ± 4.77	2.836	*P* < 0.05
	Satisfaction	16.95 ± 6.51	11.15 ± 2.62	2.125	*P* < 0.05
	Total score	80.34 ± 19.75	59.61 ± 15.14	3.911	*P* < 0.05

**Table 8:** Comparison of PAC-QOL score difference between the two groups after treatment.

Dimension	Physical conditions	Mental state	Worry about anxiety	Satisfaction	Total score
Test group	4.37 ± 1.11	8.14 ± 1.19	12.07 ± 4.58	6.45 ± 1.39	30.91 ± 8.18
Control group	2.89 ± 0.15	6.61 ± 2.62	6.92 ± 2.53	5.93 ± 2.85	22.31 ± 8.15
*T* value	3.596	1.961	5.289	0.843	4.782
*P* value	*P* < 0.05	*P* < 0.05	*P* < 0.05	*P* < 0.05	*P* < 0.05

## Data Availability

Data sharing is not applicable to this article as no data sets were generated or analyzed during the current study.
